# Determination of L-Ergothioneine in Cosmetics Based on Ultraperformance Liquid Chromatography-Tandem Mass Spectrometry

**DOI:** 10.1155/2022/4372295

**Published:** 2022-09-27

**Authors:** Li Liu, Lei Sun, Sufang Fan, Junmei Ma, Yi Wang, Qiang Li, Zhengyang Song, Yong Sun, Yan Zhang

**Affiliations:** ^1^Beijing Academy of Food Sciences, Beijing 10068, China; ^2^Hebei Food Inspection and Research Institute, Hebei Food Safety Key Laboratory, Key Laboratory of Special Food Supervision Technology for State Market Regulation, Hebei Engineering Research Center for Special Food Safety and Health, Shijiazhuang 050227, China; ^3^Department of Chemical Engineering, Key Laboratory for Industrial Biocatalysis, Ministry of Education of China, Tsinghua University, Beijing 10062, China

## Abstract

A new method was developed for the identification and determination of L-ergothioneine in cosmetics based on ultraperformance liquid chromatography-tandem mass spectrometry (UPLC-MS/MS). The pretreatment method, chromatographic column, chromatographic conditions, and mass spectrometric conditions of cosmetic samples were optimized. Methanol was chosen as the extraction solvent, 85% acetonitrile with 0.1% FA was selected as the mobile phase, and the Waters CORTECS UPLC hydrophilic interaction liquid chromatography (HILIC) column was chosen for the separation. The sample was extracted with methanol and filtered, then separated by HILIC and detected by triple-quadrupole mass spectrometry. The quantitation was done under the matrix calibration curve using the external standard method. The results showed good linear relationships in the range of 5–200 ng/mL, and the correlation coefficient was greater than 0.999 in cosmetic samples. The limit of detection was in the range of 25–50 *μ*g/kg and the limit of quantitation was in the range of 50–100 *μ*g/kg. The recoveries of the method spiked ranged from 85.3% to 96.2% and the relative standard deviation (RSD) was in the range of 0.84%–2.08% (*n* = 6). The method is simple, quick, and accurate for the determination of L-ergothioneine in cosmetics, and has great practical value.

## 1. Introduction

Ergothioneine (EGT) was originally isolated from *Claviceps purpurea* by Tanret in 1909 [1]. EGT is a naturally occurring amino acid analog that is synthesized in some bacteria and fungi but not in animals [2], which must be absorbed from food in which it is distributed very unevenly [3, 4]. L-ergothioneine (L-EGT) is the natural form of EGT. It has a high solubility in aqueous solutions and exists as a tautomer between thiol and thione forms in solution [5]. For the unique low molecular weight dietary thione, there has been a recent surge of interest in EGT [6]. EGT is a sulfur-containing amino acid analog that is well known as a potent hydrophilic antioxidant [7], meanwhile which is a biologically important compound that has been shown to be transported by the organic cation transporter novel type 1 (OCTN1) [8]. Studies on EGT had also shown that it had multiple functions in animals and humans, such as antioxidant, anti-inflammatory, antagonizing nerve damage, protecting cardiovascular, promoting reproductive health, preventing eye diseases, preventing tumors, central neurological disorders, and diabetes [9–12]. In 2017, the European Food Safety Authority (EFSA) adopted the Scientific Opinion on the Safety of L-ergothioneine, a statement on the safety of synthetic L-EGT as a novel food-supplementary dietary exposure and safety assessment for infants and young children, pregnant and breastfeeding women [13]. In recent years, EGT as a natural bioactive substance has had great application prospects in medicine, food, and health care products [14–18].

As the best known dietary sources of EGT, mushrooms and cyanobacteria have good nutritional value, medicinal value, and cosmetic value [19], mainly because their components have good antioxidant and anti-inflammatory effects [20–22], antioxidant capacity of EGT accounts for about 25% of the total antioxidant capacity of fungi extracts [23]. For the excellent free radical scavenging ability, excellent light, heat, and acid-base stability, it had shown good antioxidation, whitening [4, 24], and antiphotoaging functions when EGT was applied to cosmetics [25, 26]. Due to the excellent effect of EGT, it has become a gimmick for high-end cosmetics publicity. However, whether EGT has been added to cosmetics or not requires accurate detection methods.

Several analytical methods such as spectrophotometry, thin layer chromatography (TLC), capillary electrophoresis (CE), and high-performance liquid chromatography (HPLC) have been reported to detect EGT [2]. HPLC is the most widely used method at present. But due to the complex matrix of mushroom extracts and cosmetics, the results might be disturbed and hindered which is caused by the coabsorption of different components when using the HPLC UV-Vis detector for determination [27]. Compared with the other methods above, ultraperformance liquid chromatography-tandem mass spectrometry (UPLC-MS/MS) not only has high sensitivity and low detection limit but also has a great advantage in quantification, which can largely avoid the interference of similar components in the detection of the analyte. The determination method of EGT based on UPLC-MS/MS has great technical advantages [9].

At present, most methods focused on the determination of EGT in fungi, there were few methods for the determination of EGT in cosmetics. Therefore, the aim of this study is to develop a method for the determination of EGT in cosmetics based on UPLC-MS/MS, which will provide a reference for the determination of EGT in cosmetics.

## 2. Materials and Methods

### 2.1. Materials and Reagents

L-ergothioneine (L-EGT, purity > 98%) was purchased from Shanghai Standard Technology Co., Ltd (Shanghai, China). Acetonitrile and methanol (suitable for HPLC) were purchased from Merck (Darmstadt, Germany). Formic acid (FA) was purchased from Fisher Scientific (Loughborough, UK). Deionized water (specific resistivity was 18.2 MΩ·cm) was obtained from the Milli-Q water purification system of Millipore (Guyancourt, France). Solution A was made with deionized water introduced with 0.1% FA. Solution B was made with acetonitrile introduced with 0.1% FA.

The nylon syringe filter (0.22 *μ*m) was purchased from Agela Technologies (Tianjin, China). The toner and cream used in this experiment were purchased from local supermarkets (Shijiazhuang, Hebei, China).

### 2.2. Instruments

The Triple Quad™ 7500 QTRAP® system (SCIEX, USA) controlled by SCIEX OS software (Version 2.1.6.59781) was used for the determination of EGT. Other Instruments used in the experiment included a KQ-500E ultrasonic cleaner (Kunshan ultrasonic instrument Co., Ltd, China), a Vortex Genius 3 mixer (IKA, German), a 3-18KS centrifuge (Sigma, German), and a ME204E electronic balance (METTLER TOLEDO, USA).

### 2.3. Preparation of Standard Solutions

To prepare the stock solution of L-EGT, 10 mg (accurate to 0.0001*g*) of L-EGT was dissolved in 100 mL of deionized water. The stock solution (100 *μ*g·mL^−1^) was protected against sunlight and could be stored in a refrigerator (−20°C) for 3 months.

Dilute the stock solution 10-fold with methanol to obtain the intermediate solution. The intermediate solution (10 *μ*g·mL^−1^) was protected against sunlight and could be stored in a refrigerator (4–8°C) for 1 month.

For the preparation of the calibration curve, 1 g (accurate to 0.001*g*) of the sample was weighed in sequence into seven 15 mL graduated centrifuge tubes. 5, 10, 20, 40, 60, 100, and 200 *μ*L of intermediate solution were introduced into the tubes, followed by the other sample pretreatment steps.

### 2.4. Sample Pretreatment Method

For liquid samples, weighed 1 g of the sample (accurate to 0.001*g*) into a 15 mL graduated centrifuge tube, diluted to 10 mL with methanol, vortexed for 1 min, and extracted in ultrasonic for 10 min. After centrifugation for 5 min at a speed of 10000 rpm, the supernatant was taken through a 0.22 *μ*m nylon syringe filter for analysis.

For cream samples, weighed 1 g of the sample (accurate to 0.001*g*) into a 15 mL graduated centrifuge tube, added 10 mL of methanol, vortexed for 1 min, and extracted in ultrasonic for 10 min. After centrifugation for 5 min at a speed of 10000 rpm, the supernatant was taken through a 0.22 *μ*m nylon syringe filter for analysis.

### 2.5. Chromatography and Mass Spectrometry Conditions

The analysis was performed on a Waters CORTECS UPLC HILIC column (2.1 × 100 mm, 1.6 *μ*m). The L-EGT was eluted in an isocratic mode which was 15% solution A and 85% solution B. The flow rate is 0.4 mL·min^−1^ and the column temperature was 40°C. The injection volume was 2 *μ*L and the total analysis time was 10 min.

The mass spectrometry was run in ESI-positive mode. The spray voltage was 5500 V and the ion source temperature was 500°C. The curtain gas (CUR), nebulizer gas (GS1), and auxiliary gas (GS2) were set at 40, 35, and 70 psi, respectively, and the collision gas (CAD) was set to medium. The data were obtained in multiple reaction monitoring (MRM) mode. The entrance potential (EP) and cell exit potential (CXP) were set at 10 and 11.5 V. Other MRM parameters of L-EGT were listed in Table 1.

## 3. Results and Discussion

### 3.1. LC Column Selection

The columns used in the separation of L-EGT by HPLC included the C18 column, HILIC column, and amino column. In this study, the experiment was carried out to compare the separation effects of L-EGT on Waters XBridge BEH C18 column (2.1 mm × 100 mm, 2.5 *μ*m), Waters Acquity UPLC HSS T3 column (2.1 mm × 100 mm, 1.8 *μ*m), Waters CORTECS UPLC HILIC column (Separation on a 2.1 mm × 100 mm, 1.6 *μ*m), and Waters UPLC BEH Amide column (3.0 mm × 100 mm, 1.7 *μ*m). The results showed that the retention time on Waters XBridge BEH C18 column and Acquity UPLC HSS T3 column was short which was not conducive to the separation of impurities. And due to the high polarity of L-EGT, the mobile phase used in the separation of the two columns above had a large proportion of the aqueous phase, which was not conducive to mass spectrometry analysis. On the contrary, Waters CORTECS UPLC HILIC column and Waters UPLC BEH Amide column showed good results in retention time and the peaks were sharp in the analysis. However, due to the fact that the bonded functional groups of amino columns were likely to hydrolyze under acidic conditions, the service life of the columns was relatively short. The Waters CORTECS UPLC HILIC column was finally selected for the separation of L-EGT in this study. Extraction ion chromatography of L-EGT using different columns was shown in Figures 1∼4.

### 3.2. Mobile Phase Optimization

In this study, the methanol-water mobile phase system and the acetonitrile-water mobile phase system were compared, respectively. The results showed that the analyte in the acetonitrile-water system had a higher response in mass spectrometry analysis, but both systems had a certain tailing phenomenon. After attempting to add 0.1% FA to the mobile phase, the analyte response and peak tailing were improved. Also, the experiment compared the retention time and peak shape of the analyte under different mobile phase proportions of 80% acetonitrile, 85% acetonitrile, and 90% acetonitrile. The results showed that the peak is relatively symmetrical and the retention time could meet the requirements of separation when the mobile phase was 85% acetonitrile. Thus, 85% proportion of acetonitrile introduced with 0.1% FA was finally selected as the mobile phase. At this condition, the retention time was 5.185 min and the peak width at the base was 0.137 min, and the peak width at 50% reached was 0.037 min.

### 3.3. Optimization of Mass Spectrometry Parameters

In this study, the Electrospray ionization (ESI) mode was chosen for the determination due to the high polarity of L-EGT. The spray voltage, ion source temperature, curtain gas, ion source gas1, ion source gas2, entrance potential (EP), cell exit potential (CXP), and collision energy (CE) were optimized so that the response of precursor and product ions of L-EGT were in the suitable range.

### 3.4. Optimization of Sample Pretreatment Conditions

The HILIC column used in the experiment was sensitive to the proportion of water in the injection solution which was prone to solvent effects. Therefore, methanol and acetonitrile were initially selected as extraction solvents in the pretreatment. The extraction efficiency was compared using the two solvents and the results showed that when acetonitrile was used as the extraction solvent, cream samples were prone to agglomeration, which was not conducive to the dispersion of the sample and reduced the extraction efficiency. Thus, the experiment finally uses methanol was finally used as the extraction solvent in the pretreatment. The recoveries of extraction using methanol and acetonitrile were shown in Figure 5.

In this study, the samples were dispersed into the extraction solvent by vortex mixer and then extracted by an ultrasonic cleaner. The extraction efficiency in ultrasonic extraction was compared under 1–30 min at the concentration of 1000 *μ*g·kg^−1^, and the result showed that after 10 min of ultrasonic extraction, the concentration of L-EGT in the extract did not change significantly with the extension of the ultrasonic time. Thus, the ultrasonic extraction time was selected as 10 min. The changes in concentration under different extraction times were shown in Figure 6.

### 3.5. Linearity of Standard Curve, Limit of Detection, and Limit of Quantification

Since there were many ingredients added, the matrix of cosmetics was very complex. And the matrix effect was more obvious when using mass spectrometry. In this study, the standard calibration curve was prepared by adding a standard to the matrix sample to reduce the matrix effect and improve the detection accuracy.

The limit of detection (LOD) and the limit of quantification (LOQ) were determined at the corresponding mass concentration when the signal-to-noise ratio was 3 and 10. The LOD and LOQ of L-EGT in liquid samples were 25 *μ*g·kg^−1^ and 50 *μ*g·kg^−1^, and the LOD and LOQ in cream samples were 50 *μ*g·kg^−1^ and 100 *μ*g·kg^−1^, respectively.

The result showed a good linear relationship in the range of 5–200 ng·mL^−1^ and the correlation coefficient (*r*^2^) was greater than 0.999 as shown in Table 2.

### 3.6. Spike Recovery

Two kinds of cosmetics, cream and toner, were selected in the experiment, and L-EGT was added at three concentration levels, respectively, and the experiments were repeated 6 times for each concentration level. The spiked recoveries of L-EGT in cream samples were between 85.3% and 91.0%, and the relative standard deviation (RSD) was between 0.88% and 1.74%. The spiked recoveries of L-EGT in toner samples were between 90.3% and 96.2%, and the RSD was between 0.84% and 2.08% as shown in Table 3.

### 3.7. Stability of the Method

The interday precision was assessed by six repeated measurements of the L-EGT concentration over 6 days. For each type of sample, a positive sample was tested each day, respectively. The interday precision was determined to be within 5%, suggesting that the method provided satisfactory stability for the quantitative determination of L-EGT as shown in Table 4.

### 3.8. Determination of L-EGT in Real Samples

The developed method was used for the determination of L-EGT in real samples. Five samples of each type (cream and toner) were tested using the method, the result showed that the samples contain zero detectable concentrations of L-EGT. The method presents an easy and effective procedure for the identification and quantification of L-EGT in cosmetics samples.

## 4. Conclusions

In this study, a SCIEX Triple Quad™ 7500 QTRAP® LC-MS/MS system was used to establish a method for the determination of L-EGT in cosmetics. The experiment investigated the separation effect of different columns. The mobile phase, mass spectrometry parameters, and sample pretreatment conditions were also optimized in the experiment. The optimal procedure was taking methanol as the extraction solvent, 85% proportion of acetonitrile introduced with 0.1% FA as the mobile phase, and the Waters CORTECS UPLC HILIC column for the separation.

The results showed good linear relationships in the range of 5–200 ng/mL, and the correlation coefficient was greater than 0.999 in cosmetic samples. The LOD was in the range of 25–50 *μ*g·kg^−1^ and the LOQ was in the range of 50–100 *μ*g·kg^−1^. The recoveries of the method spiked ranged from 85.3% to 96.2% and the RSD was in the range of 0.84%–2.08% (*n* = 6).

The method was simple, fast, and accurate and could effectively avoid the interference of similar components.

## Figures and Tables

**Figure 1:** Separation effects of L-EGT on BEH C18 column.

**Figure 2:** Separation effects of L-EGT on UPLC HSS T3 column.

**Figure 3:** Separation effects of L-EGT on BEH amide column.

**Figure 4:** Separation effects of L-EGT on CORTECS UPLC HILIC column.

**Figure 5:** The recoveries of extraction using methanol and acetonitrile in cream and toner samples.

**Figure 6:** The changes in concentration under different extraction times.

**Table 1:** MRM parameters of L-EGT.

Precursor ion (*m/z*)	Product ion (*m/z*)	Collision energy (eV)	Dwell time (ms)
230.07	186.06^*∗*^	18	200
	127.01	26	200

The product ion with (^*∗*^) was used for quantification.

**Table 2:** Calibration curve, LOD, and LOQ of L-EGT.

Sample	Regression equation	Linear range/(ng/mL)	Correlation coefficient	LOD/(*μ*g/kg)	LOQ/(*μ*g/kg)
Cream	*Y* = 1.68e^5^*X*−5.11e^5^	5–200	1.000	50	100
Toner	*Y* = 2.48e^5^*X*−4.48e^5^	5–200	1.000	25	50

**Table 3:** Recovery and RSD of L-EGT (*n* = 6).

Target	Concentrations/(*μ*g·kg^−1^)	Cream		Toner	
		Recovery/(%)	RSD/(%)	Recovery/(%)	RSD/(%)
L-EGT	200	88.2	1.60	93.9	2.08
	600	88.2	1.74	91.4	0.84
	1000	90.0	0.88	92.9	1.31

**Table 4:** The stability assay of L-EGT in the cream and toner.

Sample	Mean concentrations/(*μ*g·kg^−1^)	SD/(%)	RSD/(%)
Cream	178	4.51	2.53
Toner	188	3.62	1.93

## Data Availability

The data used to support the findings of this study are available from the corresponding author upon reasonable request (snowwinglv@126.com).
